The article "Construction of Prediction Model of Deep Vein Thrombosis Risk after Total Knee Arthroplasty Based on XGBoost Algorithm" was published in 2022. Journal: Comput Math Methods Med.

# Construction of Prediction Model of Deep Vein Thrombosis Risk after Total Knee Arthroplasty Based on XGBoost Algorithm

**DOI:** 10.1155/2022/3452348

**Published:** 2022-01-25

**Authors:** Yuhuan Chen, Yingqing Jiang

**Affiliations:** Department of Orthopedics, The First Affiliated Hospital of Soochow University, Suzhou 215006, China

## Abstract

**Objective:**

Based on the XGBoost algorithm, the prediction model of the risk of deep vein thrombosis (DVT) in patients after total knee arthroplasty (TKA) was established, and the prediction performance was compared.

**Methods:**

A total of 100 patients with TKA from January 2019 to December 2020 were retrospectively selected as the study subjects and randomly divided into a training set (*n* = 60) and a test set (*n* = 40). The training set data was used to construct the XGBoost algorithm prediction model and to screen the predictive factors of postoperative DVT in TKA patients. The prediction effect of the model was evaluated by using the test set data. An independent sample *T*-test was used for comparison between groups, and the *χ*^2^ test was used for comparison between counting data groups.

**Results:**

The top five items were combined with multiple injuries (35 points), time from injury to operation (28 points), age (24 points), combined with coronary heart disease (21 points), and D-dimer 1 day after operation (16 points). In the training set, the area under the curve of the XGBoost algorithm model was 0.832 (95% CI: 0.748-0.916).

**Conclusion:**

The model based on the XGBoost algorithm can predict the incidence of DVT in patients after TKA with good performance.

## 1. Introduction

Total knee arthroplasty (TKA) is an effective method for the treatment of end-stage knee osteoarthritis, which can significantly relieve the pain in patients and promote functional recovery [1]. Deep vein thrombosis (DVT) is one of the common complications of limb fractures in the perioperative period, which can lead to pulmonary embolism and postthrombotic syndrome. The rate of sudden death caused by pulmonary embolism is as high as 34%, which seriously affects the prognosis and life of patients [2]. DVT is a venous reflux disease caused by blood coagulation in the deep vein due to various reasons. There are three factors in patients with DVT: slow blood flow, hypercoagulability, and venous wall injury [3]. Previous studies showed that the overall incidence of DVT was 69.9% per patient postoperatively [4]. Therefore, the early diagnosis and treatment of DVT are extremely important.

In recent years, the extreme Gradient Boosting (XGBoost) model has become one of the common tools for solving classification problems due to its high efficiency, flexibility, and accuracy [5]. The XGBoost model is widely used in statistics, data mining, machine learning, and artificial intelligence, because of its low input data requirements, automatic variable selection, and low computational complexity. Especially in the medical field, the XGBoost model can make use of historical case data to build models for classification and predictions [6]. Direct prediction of postoperative indicators with clinical data and specific algorithms is helpful for doctors to make reasonable and effective judgments and further guide the follow-up medical work.

The article "Construction of Prediction Model of Deep Vein Thrombosis Risk after Total Knee Arthroplasty Based on XGBoost Algorithm" was published in 2022. Journal: Comput Math Methods Med.

In recent years, a large number of studies have reported high-risk factors related to DVT [7], but there are few studies on predicting DVT after TKA by the XGBoost model. Therefore, the purpose of this study is to explore the risk factors for DVT in patients after TKA. The prediction model based on the XGBoost algorithm is aimed at providing reliable theoretical guidance for the early intervention of DVT after TKA.

## 2. Materials and Methods

### 2.1. General Information

From January 2019 to December 2020, 100 patients with TKA who met the inclusion and exclusion criteria were selected as research objects.

Inclusive criteria are patients younger than 80 years old who received unilateral TKA for the first time and without cognitive impairment and able to cooperate with the researcher and patients with stable condition at discharge without postoperative complications and who informed and agreed to participate in the study.

Exclusion criteria are patients with severe cardiovascular and cerebrovascular diseases and malignant tumors, patients with mental disorders who are unable to cooperate, patients with hip and ankle joint deformities that affect knee joint function, patients who have undergone TKA surgery or bilateral TKA surgery at the same time, and recent participants in other researches.

### 2.2. Research Queue

All patients with TKA were randomly divided into a training set (*n* = 60) and a test set (*n* = 40). The training set was used to construct the XGBoost algorithm prediction model, and the test set data was used to evaluate the prediction effect of the XGBoost model. According to the ultrasound results of both lower limbs after the operation, the patients in the training set were divided into a DVT group and a non-DVT group.

### 2.3. Indicators and Standards of Observation

Collecting baseline data include age, gender, previous medical history (hypertension and coronary heart disease), American Society of Anesthesiologists (ASA) classification, injury severity score (ISS), time from injury to operation, operation time, intraoperative blood transfusion volume, intraoperative blood loss, hemoglobin 1 day after operation, D-dimer 1 day after operation, hospital time, and combined with multiple injuries.

The article "Construction of Prediction Model of Deep Vein Thrombosis Risk after Total Knee Arthroplasty Based on XGBoost Algorithm" was published in 2022. Journal: Comput Math Methods Med.

ISS<16 is a minor injury, 16 < ISS ≤ 25 is a moderate injury, and ISS > 25 is a severe injury [8]. According to the ASA classification, patients' condition was divided into five grades: Grade I: healthy; Grade II: suffering from systemic disease, with good compensatory function; Grade III: severe systemic disease, daily functions are limited within the scope of compensation; Grade IV: compensatory function is not complete, and daily function is lost; Grade V: the condition is serious and life-threatening [9].

### 2.4. Treatment Method

The risk assessment of thromboembolism was carried out regularly for all patients after operation. To prevent DVT, patients without contraindications of anticoagulation were injected subcutaneously with low molecular weight heparin sodium 0.4 mL every day. At the same time, the plantar vein pump was performed twice a day for 20 minutes each time. One day after the operation, blood samples were collected from all patients, and the D-dimer, blood routine, and coagulation were monitored. Ultrasound examination of veins of lower limbs was performed 3-5 days after the operation. Positive patients were given low molecular heparin calcium 0.4 mL twice a day, and the plantar venous pump was stopped for DVT treatment. All patients stopped using anticoagulants 12 hours before operation and started using anticoagulants 12 hours after operation.

### 2.5. Research Outcomes and Predictors

The outcome of the study was that DVT occurred in TKA patients 3-5 days after the operation. The inner diameter of the deep vein of lower limbs was observed from bottom to top along with the operation site, and DVT was diagnosed if the following phenomena occur: The lumen below the embolic site is enlarged, and the venous lumen cannot be closed. There is a solid echo with unequal intensity in the lumen. When the occlusion is complete, pulse and color Doppler show a small amount or no blood flow signal.

### 2.6. XGBoost Algorithm Model

The XGBoost algorithm is an optimized distributed gradient computing integration algorithm. The idea of this algorithm comes from the gradient lifting iterative decision tree algorithm. Based on the gradient lifting iterative decision tree algorithm, a second-order Taylor function is added to classify the data, which is specifically completed by the following:

Goal function:

(1) $$\begin{array}{c} \frac{\wedge }{y_{i}}=\overset{K}{\underset{k=1}{\sum }}f_{k}\left(x_{i}\right),\;f_{k}\in F, \end{array}$$

where *i* = 1, 2, ⋯, *n*, *n* is the number of samples, *F* is the set corresponding to all regression trees, and *f*_*k*_ is the function in *F*.

The article "Construction of Prediction Model of Deep Vein Thrombosis Risk after Total Knee Arthroplasty Based on XGBoost Algorithm" was published in 2022. Journal: Comput Math Methods Med.

The regular term is the damage function of the model:

(2) $$\begin{array}{c} \Omega \left(f_{k}\right)=\gamma T+\frac{1}{2}\lambda {\left\|w\right\|}^{2},\;l\left(y_{i3}{\overset{\wedge }{y}}_{i}\right). \end{array}$$

The second-order Taylor function is introduced to approximately expand the loss function, and the objective function is optimized to be closer to the actual value to improve the prediction accuracy:

(3) $$\begin{array}{c} ο=l\left(y,y_{i}\;\right)+\overset{k}{\underset{k=1}{\sum }}\beta \left(f_{k}\right), \end{array}$$

where *l*(*y*, *y*_*i*_) is a model for integrating data standardization, *O* represents the difference between the predicted value of the last formula and the recorded value of the actual data, and *β* represents the normalized processing coefficient, which is used to calculate the positive value after data weighting to prevent data confusion. Formulas (1) and (2) are fused by superposition calculation of multiple data, and the predicted values of iterative samples of data are substituted into the loss function, and the calculation results are multiplied by the normalization coefficient. The final simplified formula of the XGBoost algorithm is as follows:

(4) $$\begin{array}{c} {ο}^{t}=\overset{N}{\underset{i=1}{\sum }}\left(y_{i},y^{t-1}+g_{i}f_{i}\left(x_{i}\right)+\frac{1}{2}h_{i}y_{i}\left(x_{i}\right)\right)+\beta \left(f_{i}\right). \end{array}$$

### 2.7. Statistical Methods

Single-factor analysis of variance was used to train the clinical data of the DVT group and the non-DVT group. SPSS20.0 software was used for the statistical analysis of the data. The independent sample *T*-test was used for comparison between groups, and the *χ*^2^ test was used for comparison between counting data groups.

## 3. Results

### 3.1. Process of Model Establishment

100 patients with TKA were randomly divided into the training set (*n* = 60) and test set (*n* = 40). The training set was used to construct the XGBoost algorithm prediction model, and the test set data was used to evaluate the prediction effect of the model. According to the ultrasound results of both lower limbs after operation, the patients in the training set were divided into the DVT group (*n* = 24) and the non-DVT group (*n* = 36). The predictive factors included all the items of observed indicators.  Figure 1 shows the specific modeling process.

### 3.2. Clinical Data of Patients in Training Set and Test Set

There was no significant difference between the training set and the test set in terms of gender, age, complications, ASA grade, ISS, time from injury to operation, operation time, intraoperative blood transfusion volume, intraoperative blood loss, hemoglobin 1 day after operation, D-dimer 1 day after operation, hospitalized time, and combined with multiple injuries. In addition, there was no significant difference in diabetes mellitus and hyperlipidemia, ASA grade, ISS, operation time, intraoperative blood transfusion volume, intraoperative blood loss, and hospitalized time between the DVT group and the non-DVT group. There were statistically significant differences between the two groups in terms of gender, age, hypertension, coronary heart disease, time from injury to operation, hemoglobin, D-dimer at 1 day after operation, and combined with multiple injuries (Figure 2, Table 1).

The article "Construction of Prediction Model of Deep Vein Thrombosis Risk after Total Knee Arthroplasty Based on XGBoost Algorithm" was published in 2022. Journal: Comput Math Methods Med.

### 3.3. Establishment of XGBoost Algorithm Model

By integrating the data in the training set into the XGBoost algorithm model, we have obtained important feature scoring results. The top five items were combined with multiple injuries (35 points), time from injury to operation (28 points), age (24 points), combined with coronary heart disease (21 points), and D-dimer 1 day after operation (16 points). In addition, the other three items were combined with hypertension (14 points), hemoglobin 1 day after operation (11 points), and gender (9 points), as shown in Figure 3.

### 3.4. Calibration Degree of XGBoost Algorithm Model

As shown in Figure 4, in the training set, the area under the curve of the XGBoost algorithm model was 0.832 (95% CI: 0.748-0.916).

## 4. Discussion

With the change of population structure, the number of elderly patients with TKA is increasing [10]. DVT is a common complication after orthopedic surgery. Previous studies showed that the incidence of postoperative DVT was as high as 57%-62%, and the incidence of DVT was 0.5%-44% even with routine prevention [11]. Bawa et al. showed that patients with hypercoagulability diagnoses were at a higher risk of postoperative DVT [12]. Tateiwa et al. found that the total incidence of DVT was 62.5% in 88 patients with TKA. Among the 55 patients with DVT, the incidence of distal DVT was 96.4%, and that of proximal DVT was 3.6% [13]. These results were similar to those of our study. The reason may be that TKA has caused great damage to tissues and blood vessel walls and caused more hemorrhage. In addition, patients with postoperative pain often stay in bed for braking, which further aggravates blood stasis and increases the risk of DVT. Therefore, for TKA patients, it is necessary to attach great importance to the occurrence of DVT and strengthen the screening and prevention of thrombosis.

Clinical studies have found that DVT after TKA is a risk factor for poor prognosis and death [14]. However, the risk factors leading to DVT are still inconclusive. According to the analysis of hip fracture patients, it is found that the average time interval between operation and hospitalization for patients with DVT after the operation was 9.45 days, while that for patients without DVT was 1.06 days [15]. In this study, we found that the time from injury to operation over 5 days was an independent risk factor for DVT after TKA. This result is similar to previous studies [16]. This may be due to the long-term braking, traction, or pain after the operation, which leads to prolonged stay in bed, muscle atrophy, and hypercoagulability which then leads to the formation of DVT. Therefore, patients should be admitted to the hospital as soon as possible after being injured. Surgery should be performed as soon as possible when conditions permit to reduce the risk of DVT.

The article "Construction of Prediction Model of Deep Vein Thrombosis Risk after Total Knee Arthroplasty Based on XGBoost Algorithm" was published in 2022. Journal: Comput Math Methods Med.

Patients over 60 years have decreased physical function, easily damaged intima of blood vessels, and decreased elasticity of blood vessels and blood circulation, which increases the risk of DVT. Nybo and Hvas provided that age is a risk factor for DVT [17]. Gómez-Jabalera et al. demonstrated that age over 60 years was an independent risk factor for DVT in patients after fracture operation, and it was highly specific for predicting DVT [18]. These were also consistent with our study. However, some scholars believe that the incidence of DVT has nothing to do with age. This may be due to the timely screening of DVT after injury [11]. In addition, we also found that coronary heart disease was an independent risk factor for DVT after TKA. Our results are consistent with those of previous scholars [19]. The reason may be that coronary atherosclerosis in patients with coronary heart disease leads to vascular endothelial damage, promotes platelet adhesion and aggregation, and accelerates the coagulation process, thus leading to the increased risk of postoperative DVT. D-dimer is the simplest degradation product of fibrin, and the increase of mass concentration can reflect the existence of hypercoagulability in the body, which is a nonspecific sign of thrombosis. It has been widely applied to the diagnosis and prognosis of clinical thrombotic diseases. Our study found that D-dimer was an independent risk factor for DVT after TKA, which was consistent with previous studies [20].

Davagdorj et al. built a model of noncommunicable diseases caused by smoking based on the XGBoost framework, which can realize a more accurate prediction [5]. In addition, in the diagnosis of chronic kidney disease, Ogunleye and Wang proved that the XGBoost model has a great advantage in prediction accuracy [21]. The XGBoost algorithm model established in this study has high sensitivity and specificity in predicting DVT in patients after TKA operation. Various algorithms have their own advantages and disadvantages. We will try to use new algorithms to evaluate the prognosis of the disease in the future [22, 23].

The article "Construction of Prediction Model of Deep Vein Thrombosis Risk after Total Knee Arthroplasty Based on XGBoost Algorithm" was published in 2022. Journal: Comput Math Methods Med.

There are some limitations to our study. This study was a retrospective study of a small single-center sample, which needs further verification in the prospective study of a large multicenter sample. Secondly, there are not enough influencing factors in the analysis, and there was no hierarchical analysis of these factors. In addition, although the XGBoost algorithm model has unique advantages in dealing with high-dimensional variables, complex interactions among variables, and nonlinear relationships, the effectiveness of the prediction model will also be limited by the nature, number, type, and sample of variables.

## 5. Conclusion

The model based on the XGBoost algorithm can predict the occurrence of DVT in patients after TKA with good prediction performance. The items including combined with multiple injuries, time from injury to operation, age, coronary heart disease, and D-dimer at 1 day after operation can be used as predictive indicators of DVT after TKA.

## Figures and Tables

**Figure 1:** Modeling flow chart.

**Figure 2:** Comparison of clinical data between the DVT group and the non-DVT group in the training set. There were significant differences (*P* < 0.05) between the DVT and non-DVT groups in gender (a), age (b), time from injury to operation (c), hemoglobin (d), coronary heart disease (e), and combined with multiple injuries (f).

**Figure 3:** Score of important features in XGBoost algorithm model.

**Figure 4:** The receiver operation characteristic (ROC) curves of XGBoost algorithm model.

**Table 1:** Comparison of clinical data between the DVT group and the non-DVT group in the training set 1 day after operation (mean ± SD).

Index	DVT group	Non-DVT group	*t* value	*P* value
Hemoglobin (g/L)	107.25 ± 16.33	118.39 ± 17.52	2.922	<0.05
D-dimer (mg/L)	6.24 ± 4.87	2.66 ± 3.21	4.065	<0.001

## Data Availability

The data used to support the findings of this study are available from the corresponding author upon request.
